# Reduced levels of miR‐485‐5p in HPV‐infected cervical cancer promote cell proliferation and enhance invasion ability

**DOI:** 10.1002/2211-5463.12869

**Published:** 2020-06-30

**Authors:** Yuanyuan Dai, Fengyan Xie, Yan Chen

**Affiliations:** ^1^ Department of Obstetrics and Gynecology the Third Affiliated Hospital of Wenzhou Medical University Zhejiang China

**Keywords:** cell proliferation, cervical cancer, FLOT‐1, HPV‐infected, invasion, microRNA‐485‐5p

## Abstract

Cervical cancer (CC) is the most common gynecological malignancy, with high incidence and mortality rates in China. The microRNA miR‐485‐5p has previously been reported to serve as a negative regulator of tumorigenesis in breast cancer and hepatocellular carcinoma, and miR‐485‐5p has been observed to be differentially expressed between CC and normal control tissue. Here, we confirmed that miR‐485‐5p expression is lower in CC than in adjacent normal tissue and proceeded to investigate the effects of miR‐485 on tumor behavior in CC cell lines. We report that miR‐485‐5p transcription is decreased in HPV‐infected CC tissue, and levels of miR‐485 in clinical samples are positively correlated with the 5‐year overall survival rate. The Transwell assay showed that miR‐485‐5p inhibited cell invasion and migration but had no influence on apoptosis and cell proliferation. Using a luciferase reporter assay, we demonstrated that miR‐485‐5p partially abrogated cell migration and proliferation by targeting FLOT‐1 mRNA. Transfection of HPV‐infected cervical carcinoma cells with an adenovirus vector encoding human FLOT‐1 partially diminished the inhibitory effects of miR‐485 on cell invasion. Taken, together, these data demonstrated that miR‐485‐5p suppresses the invasion of cancer cells by targeting FLOT‐1 in HPV‐infected cervical carcinoma cells.

## Graphical abstract

Inhibition of invasion and metastasis by miR‐485‐5p is dependent on direct degradation of FLOT‐1, but repression of proliferation by miR‐485‐5p is independent of FLOT‐1 in HPV‐infected cervical cancer cells.

**Abbreviations**
CC: cervical cancer
GBM: glioblastoma
miRNAs: microRNAs
MTT: 3‐(4,5‐dimethylthiazol‐2‐yl)‐2,5‐diphenyl‐tetrazolium bromide
NC: negative control
qPCR: quantitative PCR
qRT‐PCR: quantitative reverse transcriptase‐PCR
TBST: Tris‐buffered saline with Tween 20

Cervical cancer (CC) is the most common gynecological malignant tumor in developing countries [1, 2]. Although recent data suggest the relatively low incidence and mortality rates among urban residents, the burden of diseases associated with CC is still higher compared to developed countries [1]. Moreover, as a result of regional disparities in socioeconomic development, some patients cannot receive timely treatment in the early stages of tumorigenesis. Therefore, further investigation of the pathogenic mechanism and potential therapeutic targets should be a focus of gynecologists and oncologists.

MicroRNAs (miRNAs) are a class of small non‐coding RNAs that act as epigenetic regulators [3]. These molecules act by affecting a sequence of cellular and molecular mechanisms (e.g. angiogenesis, growth, differentiation, etc.) [4, 5, 6, 7, 8]. Given that the deregulation of these molecules is associated with initiation and progression of several diseases, including cancer, cardiovascular diseases, inflammatory diseases and diabetes, miRNAs might be a suitable tool for cancer diagnosis and therapy [9, 10, 11, 12]. A previous study revealed that, in gastric cancer, miR‐485 and other cancer suppressive miRNAs mapped to the 14q32.31 locus were downregulated, which enhanced the proliferation, invasion and metastasis of cancer cells [13]. miR‐485‐5p, a mature form of miR‐485, was confirmed to serve as a negative regulator of tumorigenesis in breast cancer and hepatocellular carcinoma [14, 15, 17]. The low serum levels of miR‐485‐5p were associated with poor prognosis in patients with glioblastoma (GBM) and could be considered as an independent risk factor for the prediction of survival rate [17]. In conclusion, it is widely accepted that miR‐485‐5p could exhibit a cancer suppressive effect on various kinds of malignant tumors. Although the role of miR‐485‐5p in CC is still uncertain, the results of microarray analyses have shown a differential expression of miR‐485‐5p between CC and normal control tissue [16].

The decrease of miR‐485‐5p in gastric cancer contributes to the overexpression of FLOT‐1, which leads to a decrease in cell cycle progression and consequently, in number of cells in the S phase [18, 19]. Meanwhile, the overexpression of FLOT1 was shown to promote cell invasion and metastasis, which results in poor survival. In the same study, miR‐485 was shown to target oncogenes in gastric cancer. Additionally, a recent study has demonstrated that an elevated FLOT1 expression in CC tissue facilitated lymph node metastasis [20]. Therefore, we considered that FLOT1 may be downregulated by miR‐485‐5p in CC tissue. We found that the miR‐485‐5p mimic could inhibit cell invasion and proliferation, although it had no influence on apoptosis, which explained the positive correlation between the transcriptional levels of miR‐124 with overall survival in our independent cohort of patients with CC. Our research provides a novel and promising therapeutic target for CC treatment that causes repression of cell proliferation and tumor metastasis.

## Materials and methods

### Cell culture

The primary human vaginal epithelial cells were purchased from the ATCC (https://www.atcc.org/products/all/PCS‐480‐010.aspx; catalog no. PCS‐480‐010) and were used as controls considering their similarity to cervical epithelial cells with respect to biological behavior and histological type, as reported in previous studies [21, 22, 23]. Human CC cell lines, SiHa, HeLa, Caski, C4‐1 and C‐33a, were purchased from KeLei Biotechnology Co., Ltd. (Shanghai, China) and BOSTER Biological Technology Co., Ltd. (Wuhan, China). Cells were cultured in RPMI 1640 medium supplemented with 10% fetal bovione serum (Invitrogen, Carlsbad, CA, USA), 100 U·mL‐^−1^ penicillin and 100 µg·mL^−1^ streptomycin. Cells were then incubated at 37 °C in an incubator with 5% CO_2_ and 95% relative humidity. Cells were used for subsequent experiments at a coverage rate of 80–90% after two or three passages.

### RNA extraction and quantitative PCR

For quantitative real‐time PCR, total RNA was isolated from different HPV‐infected and non‐infected fresh live cervical cells and clinical tissues using TRIzol Reagent (Invitrogen), in accordance with the manufacturer’s instructions. RNA isolated from the serum samples was extracted in accordance with previously described protocols using the Plasma/Serum Circulating and Exosomal RNA Purification Mini Kit (Norgen Biotek Corporation, Thorold, ON, Canada) [24]. We obtained 200–400 ng of eluted RNA from ~ 1000 μL of serum. Total RNA was reverse transcribed to its complementary DNA using random hexamers and Superscript III reverse transcriptase (Invitrogen) for the analysis of the transcription levels. Following reverse transcription of mRNA and miRNAs, a quantitative reverse transcriptase‐PCR (qRT‐PCR) was performed to analyze the expression of FLOT‐1 using SYBR Green PCR Master Mix (Applied Biosystems, Carlsbad, CA, USA). The sequences of the forward and reverse primers for PCR amplification of FLOT‐1 were: forward, 5'‐ACATTGCCCTGGAGACGTTAG‐3' and reverse, 5'‐ACACTGATGCCCATGTTGAC‐3', respectively. The miRNA‐485‐5p gene was analyzed by RT‐PCR, followed by qPCR analysis, as described previously [24]. The total RNA was reversely transcribed to cDNA with the TaqMan™ MicroRNA Reverse Transcription (Applied Biosystems) and a PrimeScript® mRNA cDNA synthesis kit (TaKaRa, Tokyo, Japan) and the qPCR for miRNAs was performed with the miScript SYBR Green PCR Kit (Qiagen, Shanghai, China), in accordance with the manufacturer’s instructions.

The cDNA product was amplified by PCR using SYBR Premix Ex TaqTM II (TaKaRa) and miR‐485‐5p‐ and U6‐specific primers. The primers were: miR‐485‐5p, forward, 5'‐CCAAGCTTCACCCATTCCTAACAGGAC‐3' and reverse, 5'‐CGGGATCCGTAGGTCAGTTACATGCATC‐3' (QINGKE Bio, Guangzhou, China); U6, forward, 5'‐CTCGCTTCGGCAGCACA‐3' and reverse, 5'‐AACGCTTCACGAATTTGCGT‐3'. The expression levels were normalized using GAPDH for mRNAs and U6 for miRNAs in tissue samples. miR‐16 was used as the endogenous control for the detection of miRNA levels in serum samples, as described previously [24]. Quantitative real‐time PCR data were analyzed using the $2^{-\Delta \Delta C_{t}}$ method. The results were expressed as the fold‐change over control samples, as indicated.

### Patients and tissue specimens

The study was approved by the Medical Ethics committee of the Third Affiliated Hospital of Wenzhou Medical University and we obtained the written informed consent of each patient enrolled in the study in accordance with the guidelines set by the Declaration of Helsinki. We consecutively collected and cryopreserved serum and tumor tissue samples from 78 patients with CC who had received radical hysterectomy. Out of 78 patients, 45 were diagnosed with squamous cell carcinoma. The clinical samples were obtained from The Third Affiliated Hospital of Wenzhou Medical University, and patients who had received chemotherapy and/or radiation prior to surgery were excluded from this study. The transcription levels of miR‐485‐5p were retrospectively analyzed by qPCR in serum and tissue samples. Additionally, cryopreserved tissues of 10, paired cancerous and corresponding adjacent, non‐cancerous tissue specimens were also collected for qPCR and western blotting. Follow‐up data and patient information were collected and analyzed retrospectively using medical records.

### Luciferase assay

We amplified the 3'‐UTR sequence of human FLOT1 gene from genomic DNA by PCR, cloned it into the psiCHECK vector (Promega, Madison, WI, USA) downstream of the Renilla luciferase reporter gene using standard cloning protocols. Cloned inserts were verified by DNA sequencing. The luciferase vector carrying a fragment of the 3'‐UTR of FLOT1 mRNA, which may contain the possible miR‐145 binding sites, was transfected into the CC cell line, SiHa, after treatment with oligo controls, a miR‐485‐5p mimic, or a negative control (NC) using nucleofection. After 2 days, cells were lysed and the activities of Renilla luciferase and the endogenous control, firefly luciferase, were determined using the Dual‐Luciferase Reporter Assay System (Promega). The results were normalized with firefly luciferase activity and expressed as the fold‐change over control.

### Transfections

The constructs of the pcDEF3 vector encoding human‐FLOT‐1 and GFP were purchased from the Shanghai Jikai Gene Chemical Technology Co., Ltd (Shanghai, China). The pcDEF3 vector was used for the overexpression of FLOT1 in the HPV‐infected cancer cell line, SiHa. The NC was constructed by scrambling a sequence that was incapable of encoding a target gene. Transfection was performed in accordance with the previously described standard procedure [25]. SiHa cells were seeded in 96‐well plates at a density of ~ 3000 cells per well and incubated at 37 °C. On the second day, cells were transfected with the pcDEF3 vector for 10–12 h using Lipofectamine 2000 reagent (Invitrogen), in accordance with the manufacturer’s instructions. The cells with green fluorescence indicated stable transfections with the adenoviral‐mediated vector. In total, > 85% cells with green fluorescence were detected under a fluorescence microscope, thereby indicating the successful establishment of SiHa‐NC and SiHa‐FLOT‐1 (overexpression) cell models.

### Cell apoptosis detection by flow cytometry

The apoptosis detection (Annexin FITC‐PI assay) was performed by flow cytometry as described previously with slight modification [16, 17] After transfection, cells were incubated for 48 h, followed by 24 h of treatment with 100 μm cisplatin. Cells were then harvested, washed twice with cold PBS, and then 1 × 10^6^ cells were resuspended per tube with a flow cytometry staining buffer (eBioscience, Carlsbad, CA, USA). Cells were then stained (Annexin V‐FITC/PI apoptosis detection kit; #88‐8007‐72; eBioscience) and protected from the light for 30 min. Apoptotic cells were detected by flow cytometry using BD FACSCalibur flow cytometer (BD Biosciences, Franklin Lakes, NJ, USA), and data were analyzed using flowjo, version 6.0 (https://www.flowjo.com).

### Prediction of target mRNA

According to the miRanda online website (http://www.microrna.org/microrna/home.do), we predicted the possible mRNA molecular that have potential to be target degraded by the miR‐485‐5p. The predictive score and corresponding percentile rank were used for the evaluation of binding specificity and affinity between miR‐485‐5p and the mRNA.

### Transwell assays

Transwell assays were performed to assess cell invasion using HTS Transwell‐24 system (Corning Inc., Corning, NY, USA). Cells were cultured in serum‐free RPMI 1640 medium for 24 h, followed by the addition of 100 µL of 5 × 10^4^ cells into the upper chamber, whereas the lower chamber was filled with RPMI 1640 medium supplemented with 10% fetal bovine serum as a chemoattractant. Cells from the serum‐free upper chamber have a tendency to pass through the membrane because of the presence of serum‐containing medium in the lower compartment, which allowed the estimation of cell migration and invasion ability. After incubation at 37 °C for 24 h, cells in the lower compartment that had passed through the membrane were stained with Giemsa, fixed with 4% paraformaldehyde on the slides and then counted under a light microscope.

### Western blotting

Total protein was isolated from cells of cervical para‐carcinoma or cancerous tissues by the RIPA lysis buffer and denatured by high‐temperature water bath. Equivalent protein lysates were separated by 10% SDS/PAGE gel electrophoresis and then transferred to nitrocellulose membranes. The membranes were first blocked with 5% (w/v) dried skimmed milk in Tris‐buffered saline with Tween 20 (TBST) for 1 h at 25 ± 2°C and then probed with the indicated primary antibodies (dilution 1 : 3000; anti‐human FLOT‐1 antibody; Abcam, Cambridge, MA, USA) overnight at 4 °C. Subsequently, the membranes were washed three times with 1 × TBST followed by incubation with the corresponding horseradish peroxidase‐conjugated secondary antibodies for 2 h at room temperature. GAPDH (anti‐GAPDH from Kangcheng, Inc., Shanghai, China) was used as an internal control. After washing three times with TBST, the protein bands were detected by an enhanced chemiluminescence system (Pierce Biotechnology, Rockford, IL, USA) using Alpha Innotech FluorChem SP (San Leandro, CA, USA).

### Cell proliferation and migration assays

The proliferation of HPV‐infected or non‐HPV‐infected cell lines *in vitro* was determined by the 3‐(4,5‐dimethylthiazol‐2‐yl)‐2,5‐diphenyl‐tetrazolium bromide (MTT) assay using the Vybrant MTT Cell Proliferation Assay Kit (Invitrogen), in accordance with the manufacturer’s instructions. Wound healing assays were performed as described previously [26]. HPV16‐infected cell lines and non‐HPV‐infected cell lines were incubated in serum‐free medium for 48 h. A linear wound was then gently introduced in the center of the cell monolayer using a 200‐μL tip, and cells were then subjected to stimulation with high glucose for 24 h and dynamic observation for a further 24 h. Images were then captured using an IX 71 microscope (Olympus, Tokyo, Japan).

### Statistical analysis

All experiments were repeated at least five times and the data are reported as the mean ± SEM. Unpaired *t*‐tests were used to determine the statistical differences between the two groups in each analysis. ANOVA was used for the comparison of multiple groups over two groups. The Student–Newman–Keuls test was used for pairwise multiple comparisons test among multiple groups *P < *0.05 was considered statistically significant. Overall survival was defined as the time from diagnosis to the date of cancer‐related death during the follow‐up period, and progression‐free survival was defined as the time from receiving surgery treatment to the onset of recurrence during the follow‐up period. After determining cut‐offs using cutoff finder (http://molpath.charite.de/cutoff), survival curves were plotted using the Kaplan–Meier method and analyzed by the log‐rank test. All statistical analyses were performed using spss, version 13.0 (SPSS Inc., Chicago, IL, USA).

## Results

### The expression levels of miR‐485‐5p were decreased in HPV‐infected cervical cancer cell lines and tumor tissue samples

To confirm the differential transcriptional levels of miR‐485‐5p between cancer tissue and normal cervical tissue, we performed a qRT‐PCR to examine the expression of miR‐458‐5p between CC tissue and adjacent, non‐cancerous tissue from the same individual. We found that the expression of miR‐485‐5p was significantly decreased in cancer tissue compared to non‐cancerous tissue (Fig. 1A). To further investigate this differential expression, various CC cell lines, including HPV‐infected and non‐HPV‐infected cell lines, were investigated for the expression of miR‐485‐5p and compared to the expression of miR‐485‐5p in HCerEpiC cells. We found a significant decrease in miR‐485‐5p levels in the cell lines, including HeLa, SiHa, Caski and C4‐1 cells, whereas, in the C33A cell line, the expression level of miR‐485‐5p remained unaltered (Fig. 1B). Furthermore, in the HPV16‐infected cell lines, SiHa and Caski, we unexpectedly found that miR‐485‐5p expression levels were significantly down‐regulated compared to the levels of miR‐485‐5p in HPV18‐infected cell lines. However, no difference was observed between cell lines infected with the same strain of HPV. This result suggests that the HPV‐infection may be the indispensable, vital factor contributing to the reduced expression of miR‐485. Transcription factors, which could possibly be activated by viral sequence integration, impede miR‐485‐5p expression by possibly binding to the specific promoter that controls its transcription, influencing the initiation of transcription.

**Fig. 1:** Differential expression levels of miR‐485‐5p in normal cervical tissue and CC. (A) Differential expression levels of miR‐485‐5p between adjacent, non‐cancerous and cancerous tissue, measured by qRT‐PCR. The specimens were obtained from five patients with cervical squamous carcinoma. Error bars represent the SD. (B) Differential expression levels of miR‐485‐5p between human ectocervical‐vaginal epitheilum cells and various CC cell lines, including HeLa, SiHa, Caski, C4‐1 and C33A. Data are representative of the mean values of five independent experiments and the SEM of five replicates. Statistical analyses were performed using Student’s *t‐*test for single comparisons, *n* = 5. Error bars represent the SD. *P < 0.05, **P < 0.01.

### The low expression levels of miR‐485‐5p were associated with poor overall survival and reduced progression‐free survival

To investigate the correlation between transcription levels of miR‐485‐5p and survival in CC patients, we determined the transcription levels of miR‐485‐5p in CC tissue and compared them with that of normal, para‐carcinoma tissue as a reference in our dependent patient cohort, which includes 78 patients with CC. In Fig. 2A, the results are presented as the fold‐change in miR‐485‐5p expression level in CC tissues, such as squamous carcinoma, adenocarcinoma and mixed carcinomas of the cervix, compared to normal para‐carcinoma tissue. The different pathological types had similar miR‐485‐5p transcription levels (Fig. 2A). The cut‐off value for miR‐485‐5p fold‐change was determined using cutoff finder. By survival curve analysis and the log‐rank test, we confirmed that the lower expression levels in cancer tissue had adverse effects on progression‐free survival (*P* = 0.02) (Fig. 2C), although they had no effect on the 1‐year overall survival rate (*P* = 0.27) (Fig. 2B). We also determined the serum levels of miR‐485‐5p in patients, including patients with all CC pathological types. However, we did not identify any relationship between the serum levels of miR‐485‐5p and overall survival (*P* = 0.35) (Fig. 2D) or progression‐free survival (*P* = 0.41) (Fig. 2E).

**Fig. 2:** Correlation between patient prognosis and expression levels of miR‐485‐5p in serum and cancerous tissue. (A) Expression levels of miR‐485‐5p in various pathological types of CC tissues compared to the normal, para‐carcinoma tissues. Specimens were obtained from 78 patients with CC, most of whom were diagnosed with squamous carcinoma. Statistical analyses were performed using ANOVA for comparison of multiple groups. SCC, *n* = 45; AC, *n*‐12; Mixed, *n* = 21. Error bars represent the SD. (B, C) Overall survival and progression‐free survival in patients with higher and lower expression levels in cancerous tissues according to survival analysis. No statistical difference was observed in overall survival between the two groups, *n* = 78. (D, E) Overall survival and progression‐free survival in patients with higher and lower serum expression levels. No statistical difference was observed in overall survival and progression‐free survival between the two groups. Survival curves were plotted by the Kaplan–Meier method and a log‐test was used to calculate the statistical significance, *n* = 78. Error bars represent the SD.

### The targeted reduction of FLOT‐1 by miR‐485‐5p mimics repressed cell invasion and metastasis

Previous studies have demonstrated that the elevated expression of FLOT‐1 augments invasion and migration by regulating NF‐κB and Wnt/β‐catenin‐induced epithelial‐mesenchymal transition. However, the upstream regulatory mechanism leading to the overexpression of FLOT‐1 was not identified. We considered the downregulation of miR‐485‐5p to be the critical factor that leads to the ectopic expression of FLOT‐1 and the activation of the downstream signaling pathways associated with tumor invasion and metastasis. We found significantly reduced expression of FLOT1 in CC tissue compared to para‐carcinoma tissue (Fig. 3A,B). Furthermore, the negative correlations between serum levels or expression *in situ* of miR‐485‐5p and expression of FLOT1 in CC tissue were identified according to linear correlation analysis (Fig. 3C,D). Then, we hypothesized that the degeneration of FLOT‐1 mRNA is caused by binding of the small non‐coding RNA, miR‐485‐5p, to its 3'‐UTR region, and reduced miR‐485‐5p expression in CC cell lines represses this deterioration. To address this hypothesis, we performed luciferase assays, in which a fragment of the 3'‐UTR of FLOT‐1 mRNA was cloned into the psiCHECK vector. We identified the predicted miRNA response elements within the 3'‐UTR of FLOT‐1 mRNA for binding of miR‐485‐5p (Fig. 4A). Initially, we identified the transfection efficiency of mimic or inhibitor. We found that the application of mimic or inhibitor would obviously alter the expression of miR‐485‐5p (Fig. 4B). As expected, the miR‐485‐5p mimic inhibited luciferase activity in HPV16‐infected cell lines (Fig. 4C) and reduced the expression of FLOT‐1, whereas inhibitor increased the expression of FLOT‐1 (Fig. 4D). To further investigate the regulatory effect of miR‐485‐5p, the expression of FLOT‐1 was determined in non‐HPV‐infected cell lines by a quantitative real‐time PCR and it was found that FLOT‐1 expression remained unaltered in non‐HPV‐infected CC cell lines after administrated by miR‐485‐5p mimic or inhibitor (Fig. 4D), which was consistent with the previous results indicating unchanged expression levels of miR‐485 in both normal cervical epithelial cells and non‐HPV‐infected cell lines. This illustrated that miR‐485‐5p exhibits no effect on FLOT‐1 expression in non‐HPV‐infected cell lines. The alterations of FLOT‐1 expression after treated by mimic or inhibitor in HPV‐infected cells were verified by immunoblot assays (Fig. 4E). Based on a previous study demonstrating that an elevated expression of FLOT‐1 promoted cancer cell invasion and metastasis, we confirmed the effect of miR‐485‐5p on cell invasion and migration in HPV16‐infected and non‐HPV‐infected cell lines. We found that the miR‐485‐5p mimic attenuated but inhibitor aggravated the metastatic and invasive potential of HPV16‐infected cells, although it had no influence on non‐HPV‐infected cells (Fig. 4F,G). This confirmed that the miR‐485/FLOT‐1 axis regulates tumor invasion and metastasis only in HPV‐infected cell lines.

**Fig. 3:** Expression of FLOT‐1 in CC tissue and the correlation between the expression of FLOT1 and miR‐485‐5p. (A) Significantly reduced expression of FLOT‐1 in the cancerous tissue compared to paired para‐carcinoma tissue in different subtypes of cervical carcinoma measured by an immunoblot assay. Data are representative of the mean values of five independent experiments (*n* = 5) and the SEM of five replicates. The statistical test used *t*‐test methods. *P < 0.05, **P < 0.01. (B) Expression of FLOT‐1 in the cancerous tissue compared to paired para‐carcinoma tissue in different subtypes of cervical carcinoma as measured by qRT‐PCR. The statistical test used *t*‐test methods, *n* = 5, *P < 0.05, **P < 0.01. (C) Linear correlation between the expression of FLOT1 and miR‐485‐5p in CC tissue from 45 SSC patients, *n* = 45. *P* < 0.05 indicates statistical significance. (D) Linear correlation between the expression of FLOT1 in the CC tissue and expression levels of miR‐485‐5p in the serum samples from 45 SSC patients, *n* = 45. *P* < 0.05 indicates statistical significance.

**Fig. 4:** miR‐485‐5p reduced the invasion and metastasis by targeting degradation of FLOT‐1. (A) Predicted miRNA response elements within the 3'‐UTR of FLOT‐1 specific for miR‐485‐5p and the relative score that reflected the ability of specific binding. (B) Application of mimics significantly promoted the expression of miR‐485‐5p measured by RT‐PCR and inhibitors significantly repressed the expression of miR‐485‐5p. (C) Luciferase activity was detected by the dual‐luciferase reporter assay in SiHa cells. (D) Introduction of miR‐485‐5p mimic reduced and inhibitor increased significantly the expression of FLOT‐1 determined by a quantitative real‐time PCR in the HPV‐infected cell line, SiHa, although it had no influence on FLOT‐1 expression in the non‐HPV‐infected cell line, C33A. (E) Immunoblot assay and its quantitative analysis. The results of immunoblot assay demonstrated that the introduction of miR‐485‐5p mimic and inhibitor reduced and increased, respectively, the expression of FLOT‐1 in the HPV‐infected cell line, SiHa. (F) Representative Transwell assays performed to determine the number of cells that migrated into the lower chamber when comparing a NC and miR‐485‐5p mimic or an inhibitor‐treated group in the HPV‐infected and non‐HPV‐infected cell lines. Quantitative analysis of cells in the lower chamber is based on five independent experiments in the HPV‐infected cell line, SiHa scale bars = 100  µm. (G) Representation of migration distance difference between NC and miR‐485‐5p mimic or inhibitor‐treated groups in HPV‐infected and non‐HPV‐infected cell lines. Quantitative analysis is based on five independent experiments in the HPV‐infected cell line, SiHa. Migration distance was significantly decreased compared to the group that was not treated with the mimic. Scale bars = 100  µm. Data are representative of the mean values of five independent experiments and the SEM of five replicates. ANOVA and the Student–Newman–Keuls test was used for comparisons of multiple groups in (B) to (D). *P < 0.05, **P < 0.01. Statistical analyses were performed in (E) to (F) using Student's *t*‐test for single comparisons, *n* = 5. *P < 0.05, **P < 0.01.

### The miR‐485‐5p mimic abrogated the proliferation of HPV16‐infected cervical carcinoma cells, independently of FLOT‐1 downregulation

The MTT assay was used to assess the proliferative ability of HPV16‐infected and non‐HPV‐infected CC cell lines after treatment with miR‐485‐5p. We found that miR‐485‐5p repressed the proliferation of HPV‐infected cell lines (Fig. 5A). However, it had no influence on the proliferation of non‐HPV‐infected cervical carcinoma cell lines (Fig. 5B). The transfected efficiency of scramble and FLOT‐1 overexpression groups based on the GFP fluorescence is presented in Fig. 5C. We transfected HPV‐infected cell lines with pcDEF3 vector encoding human FLOT‐1 protein, simultaneously treating them with the miR‐485 mimic. The additional introduction of the exogenous gene increased the expression of FLOT‐1, although cell proliferation was still reduced in HPV‐infected cell lines (Fig. 5D,E), demonstrating that the downregulation of cell proliferation by miR‐485 for HPV‐infected cell lines may be independent of the degradation of FLOT‐1 mRNA. These results suggested that miR‐485‐5p may have multiple gene targets regulating the behavior of tumors.

**Fig. 5:** miR‐485‐5p had a negative influence on cell proliferation independent of the expression of FLOT‐1 in HPV‐infected cell lines. (A, B) Cell proliferation evaluated by the MTT assay in HPV‐infected and non‐HPV‐infected cell lines. Measuring the optical density in the MTT assay showed that miR‐485‐5p significantly inhibited the growth of SiHa compared to the control group. miR‐485 had no influence on the cell proliferation of non‐HPV‐infected cell lines. (C) Representative results for transfection of pcDEF3 vector encoding human‐FLOT‐1 and GFP indicating the expression of GFP in transfected cells by a contrast (upper) and fluorescence (lower) microscopy. Scale bars = 100 µm. (D) Exogenous introduction of adenoviral vector encoding FLOT‐1 increased the expression of FLOT‐1, as determined by a qRT‐PCR assay. (E) Exogenous introduction of adenoviral vector encoding FLOT‐1 had no influence on cell proliferation of the SiHa cell line. Data are representative of the mean values of five independent experiments and the SEM of five technical replicates. Statistical analyses were performed using Student's *t*‐test for single comparisons, *n* = 5. *P < 0.05, **P < 0.01.

### The miR‐485‐5p mimic had no influence on cisplatin‐induced apoptosis in various cervical cancer cell lines

Because miR‐485‐5p regulates multiple targets, we hypothesized that miR‐485‐5p may have widespread effects on the ability of tumor cells to overcome resistance to apoptosis and sensitivity to chemotherapy, both of which the aim of most cancer therapies. Hence, the effect of a miR‐485‐5p mimic on apoptosis was also examined by flow cytometry. We found that the miR‐485‐5p mimic had no influence on apoptosis induced by chemotherapy, regardless of the type of cell lines (Fig. 6A,B). These results demonstrated that miR‐485‐5p had a negative effect on proliferation, metastasis and invasion, whereas it had no effect on apoptosis or sensitivity to chemotherapy in HPV‐infected cell lines.

**Fig. 6:** miR‐485‐5p had no influence on apoptosis in HPV‐infected cell lines. (A) Representative flow cytometry analysis. Annexin‐V and propidium iodide (PI) staining was used to assess the apoptosis rate. The results were analyzed using flowjo, version 7.0. The scatter plots contain both PI and Annexin‐V channels. SiHa and C33A cells treated with cisplatin (100 µm) were used for the detection of apoptosis rate after introduction of the miR‐485‐5p mimic. (B) Quantitative analysis of early and late apoptosis rates by flow cytometry in cisplatin‐induced SiHa and C33A cells pre‐treated with mimic or control oligo. No statistically significant difference was observed with respect to early or late apoptosis rates.

## Discussion

Small non‐coding RNAs such as miR‐485‐5p can regulate gene expression at the transcription level by targeting and degrading the specific mRNAs. It has been reported that numerous miRNAs have different and significant effects on the regulation of malignancy‐related processes, including proliferation, apoptosis, invasion and metastasis, by negatively regulating oncogenes or tumor suppressor genes. Therefore, further research into the underlying mechanism of the aberrant transcriptional regulation is critical for understanding oncogenes and identifying novel therapeutic targets [11, 27, 28, 29].

A previous study confirmed that FLOT‐1 could promote the invasion and metastasis of CC cell lines by activating the NF‐κB and Wnt/β‐catenin pathways [20], and the expression levels of FLOT‐1 were positively correlated with poor prognosis [20]. The present study demonstrated FLOT‐1 to have an adverse effect on survival by accelerating lymph node metastases in CC. However, the transcriptional regulation mechanism of FLOT‐1 in CC was not determined. Additionally, in other investigations of tumor invasiveness, the role of FLOT‐1 with respect to promoting more aggressive behaviors has been confirmed. The targeted upregulation of FLOT‐1 and CAV1 attributed to a decrease in miR‐124 level in clear cell renal cell carcinoma and increased cancer cell proliferation, invasion and metastasis in *in vitro* assays. The overexpression FLOT1 and CAV1 altered the proportion of cells in the S phase of the cell cycle [30]. In addition, miR‐506 was reported to be downregulated in renal cancer cell lines and clear cell renal cell carcinoma specimens, and its overexpression was shown to inhibit cell growth and metastasis, whereas exogenous introduction of FLOT‐1 along with miR‐506 mimics abrogated rescued tumor behavior. Meanwhile, the high expression of FLOT‐1 has shown to have adverse effects on hepatocellular carcinoma survival by accelerating cancer progression [31]. The effects of FLOT‐1 in other malignant tumors, such as breast cancer and nasopharyngeal carcinoma, have also been determined [32]. Our results demonstrated that FLOT‐1 could be considered as an oncogene playing an important role in accelerating cancer progression, mainly by affecting invasion and metastasis. More importantly, the clinical prognosis is correlated with the expression of FLOT‐1 in cancer tissue [20], which suggests that the degeneration and downregulation of FLOT‐1 could be considered as potential therapeutic strategies for controlling malignant tumors.

The small non‐coding RNA, miR‐485‐5p, has been regarded as an important molecule in various types of carcinomas. miR‐485‐5p was mapped to the 14q32.31 locus with a sequence alignment tool using the GenBank database (https://www.ncbi.nlm.nih.gov/genbank), and it represses cell proliferation and the invasion of hepatocellular carcinoma by targeting degeneration of stanniocalcin [15]. Lou *et al*. [14] have reported that miR‐485‐3p and miR‐485‐5p suppress mitochondrial respiration to attenuate metastasis in breast cancer. In lung adenocarcinoma, miR‐485‐5p was shown to inhibit metastasis by blocking epithelial–mesenchymal transitions [33]. Targeting FLOT‐2 degeneration was revealed to be the underlying mechanism involved in the regulation of miR‐485‐5p in lung adenocarcinoma [34]. Moreover, the serum levels of miR‐485‐3p have been shown to have positive influences on the cell survival in GBM. Recently, Wang *et al*. [24] performed microarray‐based detection to identify differential miRNA profiles in the sera from patients and healthy individuals. Five‐year overall survival and progression‐free survival were significantly improved in patients with GBM showing high serum levels of miR‐485‐3p [24]. It has been reported that the transcription levels of some miRNAs located at 14q32.31, including miRNA‐485, miR‐154 and miR‐299‐5p, were significantly decreased in metastatic prostate cancer. The specific region in chromosome 14 contains numerous cancer‐related miRNAs sequences, for which downregulation is associated with malignant cell behaviors, such as proliferation, apoptosis, invasion and metastasis. Therefore, the miR‐485 may be a vital suppressive molecule in tumorigenesis and cancer progression [13].

We initially selected some miRNAs based on previously published microarray results. We found statistically significant differences in the expression levels of miR‐485‐5p in CC tissues compared to those in adjacent, non‐cancerous tissues [16]. Because the target of miR‐485‐5p in CC remained undiscovered, we used an online miRNA target and expression database (http://www.microrna.org/microrna/home.do) to identify potential target genes that could possibly influence tumor invasion and metastasis. Furthermore, we recognized a correlation between miR‐485‐5p and FLOT‐1 expression, which was shown in a previous study in gastric cancer. The study shows that miR‐485 targets FLOT‐1 to reduce its expression, altering the malignant phenotype of gastric cancer cells by affecting their invasion and migration. Furthermore, the role of FLOT‐1 in promoting lymph node metastasis in CC has been confirmed in another previous study [20]. However, the role of miR‐485/FLOT‐1 axis in CC was unknown. Therefore, we analyzed the effects of miR‐485‐5p on the behavior of tumor cells in CC. Experiments were performed using HPV‐infected and HPV‐negative cell lines. We found that the dysregulation of miR‐485‐5p only emerged in the HPV‐infected cell lines, most significantly in the HPV16‐infected cell lines. As noted in a previous study [35], HCV‐infection would have an obvious influence on the microRNA expression profile of hepatocellular carcinoma tissue, which resulted in the activation of signaling pathways involved in the immune response and oncogene regulation. In patients with chronic viral hepatitis, disease progression is associated with the activation of miRNA pathways that promote cell proliferation and fibrogenesis but preserve the differentiated hepatocyte phenotype [36]. These studies demonstrate that the viral infection indeed leads to the change of expression profile of microRNA, which further has an adverse influence on the physiological homeostasis. The dysregulation of microRNA after viral infection would promote tumorigenicity and lead to more invasive biological behaviors. This finding might have been determined by the integration of viral genome sequence into sites where the gene encodes transcription factors regulating the production of pre‐miR‐485, as described previously [37]. HPV genomes were significantly enriched near specific integration breakpoints, indicating that fusion between viral and human DNA may have occurred in the host cancerous cells. Therefore, we hypothesized that the HPV integration‐driven cervical carcinogenesis could be attributed to the dysregulation of microRNA or other trans‐acting factors as presented in the present study.

## Conclusions

Our data have demonstrated that miR‐485‐5p might target the degradation of FLOT1 mRNA in CC, and the deficiency of miR‐485‐5p may contribute to the more aggressive malignant phenotype, which includes an increase in cancer cell proliferation, invasion and metastasis. FLOT‐1 was likely not the only target of miR‐485‐5p because the negative regulation of cell proliferation by miR‐485‐5p was independent of FLOT‐1 expression. Our results highlight a novel, potential therapeutic target for CC.

## Conflict of interest

The authors declare no conflict of interest.

## Author contributions

YD and YC conceived the study and designed the experiments. YD, FX and YC contributed to the data collection, performed the data analysis and interpreted the results. YD wrote the manuscript. YC contributed to the critical revision of article. All authors read and approved the final manuscript submitted for publication.
